# Analysis of Efficacy, Complications, and Inflammatory Reactions of Bridge Combined Internal Fixation System for Periarticular Fractures of the Shoulder

This article has been retracted.

**DOI:** 10.1155/2022/5048172

**Published:** 2022-08-21

**Authors:** Haiyun Xu, Youliang Fan, Jiajun Lu, Yixiong Wu, Xiaoguang Feng

**Affiliations:** Department of Orthopedics, The Fourth People's Hospital of Changzhou, Changzhou, 213100 Jiangsu, China

## Abstract

**Objective:**

The aim of the present research is to analyze the impact of the bridge combined internal fixation system (BCFS) on efficacy, complications, and inflammatory reactions of periarticular fractures of the shoulder.

**Methods:**

A retrospective analysis was performed on 100 patients with periarticular fractures of the shoulder admitted between January 2016 and January 2020. Patients were assigned to the observation group (OG) and control group (CG) according to different treatment schemes, with 50 cases in each group. Patients in OG were intervened by BCFS, while those in CG were routinely given plate fixation. The treatment outcome, complications, and inflammatory reaction of the two groups were compared.

**Results:**

The results showed better treatment outcome, shoulder joint function recovery, and inflammatory reaction alleviation of OG compared with CG. Besides, statistically shorter fracture healing and hospitalization time as well as fewer complications were determined in OG.

**Conclusion:**

These results demonstrate that compared with the plate fixation system, BCFS can significantly improve the surgical efficacy and healing efficiency and alleviate the inflammatory response of patients, with a low complication rate, all of which contribute to faster recovery of periarticular fractures of the shoulder. Hence, BCFS is an ideal choice for periarticular fractures of the shoulder that deserves clinical promotion.

## 1. Introduction

Fractures are common injuries that occur at all ages, usually triggered by collisions, stress, or diseases [1]. As a kind of fractures, periarticular fractures of the shoulder joint include clavicle and scapula fractures, fractures of the upper end of the humerus and of the outer clavicle with coracoclavicular ligament rupture, displaced fractures of the outer 1/3 of the clavicle, open fractures, and fractures combined with vascular and nerve injuries, usually requiring surgical treatment [2]. However, fracture healing, a complex process that takes time, is affected by the blood supply, bone stability, and inflammation at the fracture site [3]. Besides, improper fixation material selection or inadequate fixation adversely influences functional recovery and fracture healing of the affected limb [4]. According to relevant epidemiological data, about 4.3% of the elderly in the United States have another shoulder fracture within one year after surgery [5]. Therefore, this study starts with the fixation of the periarticular fracture of the shoulder, aiming at finding a more ideal treatment.

Internal fixation is currently the major surgical treatment for fractures [6], which has been shown to prompt patients to regain their mobility and reduce the occurrence of serious complications [7]. When dealing with different clinical types of fractures, choosing an appropriate internal fixation method to maximize patients' recovery has become the key to clinical work [8]. The bridge combined fixation system (BCFS), a novel type of internal fixation device independently developed by Professor Xiong Ying from Yan'an Hospital affiliated to Kunming Medical University [9], has the advantages of small volume, firm fixation, simple operation, few postoperative complications, and promising clinical application potential [10]. Guo et al. [11] reported that BCFS is effective and safe for severe comminuted femoral fractures.

At this stage, BCFS is primarily used in the treatment of pelvic and femoral fractures, but little is known regarding its application in periarticular fractures of the shoulder. Accordingly, this paper mainly discusses the efficacy, complications, and inflammatory reactions of BCFS in the treatment of periarticular fractures of the shoulder, hoping to provide a new reference for the management of such fractures.

## 2. Data and Methods

### 2.1. General Data

This retrospective study selected 100 patients with periarticular fractures of the shoulder treated between January 2016 and January 2020. According to different fixation schemes, 50 patients treated with BCFS were set as the observation group (OG), and another 50 cases with routine plate fixation were used as the control group (CG). CG comprised 28 males and 22 females whose age range was (37.06 ± 9.14) years old; the fractures were attributed to car accidents in 22 cases, falls in 11 cases, crushes in 12 cases, and others in 5 cases. In OG, the male-female ratio and age range were 31 : 19 and (37.32 ± 8.47) years old, respectively, and the causes of injuries were car accidents in 18 cases, falls in 16 cases, crushes in 5 cases, and others in 11 cases. The two cohorts of patients were clinically comparable with no statistical difference in sex, age, cause of injury, and other baseline data (*P* > 0.05). This research was conducted after obtaining approval from the Ethics Committee of the Fourth People's Hospital of Changzhou and informed consent from patients and their families.

### 2.2. Eligibility Criteria

Inclusion criteria were as follows: diagnosis of periarticular fractures of the shoulder by clinical X-ray examination, age: 20-65, no relevant history of periarticular fractures of the shoulder, informed consent provided, and active cooperation with the study.

Exclusion criteria were as follows: old fractures or pregnant/lactating women; diseases of vital organs, clotting disorders, or inability to tolerate surgery; severe mental illness; inconsistency with the inclusion criteria; and uncooperative patients or those with defective case records that affected the curative effect judgment.

### 2.3. Treatment Methods

CG (plate fixation group) was as follows: plate fixation was used to treat patients in this group. The patient was placed in the lateral decubitus position for general anesthesia and routine disinfection. After incision, a 6-8-hole steel plate was used for fixation, and routine orthopedic nursing was performed postoperatively.

OG (BCFS group) was as follows: patients in this study were treated with BCFS. The patient's posture, anesthesia, disinfection, and postoperative care were all consistent with those of CG. Attention was paid to protecting important nerves and blood vessels during the operation. The fixation rod was then remodeled according to the fracture site and shape, and the appropriate fixation position was selected by rotating and sliding the connecting block on the fixation rod to ensure the fixation effect.

### 2.4. Efficacy Assessment

Marked effectiveness: the function of the affected limb returned to normal, with pain disappeared, anatomically reduced fracture, and well aligned fracture showed by X-ray film

Effectiveness: the function of the affected limb basically returned to normal, with basically disappeared pain, reduced fracture, and X-ray indicating over 1/3 alignment of the fracture

Ineffectiveness: the function of the affected limb has not returned to normal, with no reduction of the fracture or slow healing and even the occurrence of other complications

### 2.5. Endpoints

1. Curative effect: please refer to efficacy assessment for the evaluation standard of curative efficacy. The overall response rate (ORR) is the percentage of the sum of markedly effectiveness+effectiveness cases in all cases
2. Clinical indices: clinical indices (fracture healing time and length of hospital stay [LOS]) were recorded
3. Complication rate: complications, including healing deformity, blood ooze, and infection, were observed and recorded during postoperative recovery
4. Shoulder joint function score: the Constant-Murley Scale (CMS; score range: 0-100 points) was used before and 6 months after operation, assessing patients' shoulder joint function from pain (15 points), shoulder joint mobility (40 points), power (25 points), and activity of daily living (ADL; 20 points), with higher scores indicating better shoulder joint function
5. Serum inflammatory indicators: serum was extracted, and enzyme-linked immunosorbent assay (ELISA) [12] was utilized to test pre- and posttreatment alterations of serum inflammatory factors like tumor necrosis factor *α* (TNF-*α*), interleukin (IL)-1*β*, and IL-6. The operation steps strictly followed human TNF-*α*, IL-1*β*, and IL-6 ELISA kits supplied by Wuhan Fine Biotech

### 2.6. Statistical Processing

SPSS 21.0 (SPSS, Inc., Chicago, IL, USA) and GraphPad Prism 6 (GraphPad Software, San Diego, USA) were responsible for data analysis and visualization, respectively. *P* < 0.05 was supposed to indicate statistical significance. The *χ*^2^ test was used for intergroup comparisons of enumeration data (sex, age, etc.) represented by number of cases/percentage (*n*/%). For the quantitative data (mean age, fracture healing time, etc.) given mean ± SEM, independent sample *t*-test and paired *t*-test were employed for between-group and within-group comparisons, respectively.

## 3. Results

### 3.1. Baseline Data of Patients with Periarticular Fractures of the Shoulder

The analysis of patients' general data (Table 1) revealed comparability between the two groups, as no statistical difference was found in sex, age, average age, cause of injury, education level, drinking history, place of residence, marital status, etc. (*P* > 0.05).

### 3.2. Clinical Indices of Patients with Periarticular Fractures of the Shoulder

We recorded patients' fracture healing time and LOS to compare and analyze the influences of the two fixation methods on the clinical indices of patients with periarticular fractures of the shoulder (Table 2). It was found that the fracture healing time and LOS were statistically shorter in OG versus CG (*P* < 0.05).

### 3.3. Curative Effect of Patients with Periarticular Fractures of the Shoulder

We analyzed patients' outcomes to assess the impacts of the two treatments on patients with periarticular fractures of the shoulder (Table 3). Data showed an ORR of 96.00% in OG and 80.00% in CG, with statistical significance (*P* < 0.05).

### 3.4. Complication Rate in Patients with Periarticular Fractures of the Shoulder

By comparing and analyzing the incidence of complications in terms of healing deformity, blood ooze, and infection (Table 4), we found that the total complication rate was statistically lower in OG compared with CG (4.00% vs. 22.00%, *P* < 0.05).

### 3.5. Patient's Shoulder Joint Function Scores

We recorded the shoulder joint function (CMS) scores before and 6 months after operation (Figure 1). Data showed no statistical difference in pretreatment CMS scores between the two groups (*P* > 0.05); the posttreatment scores elevated in both cohorts (*P* < 0.05), and the improvement degree of shoulder joint function was more obvious in OG (*P* < 0.05).

### 3.6. Serum Inflammatory Indicators (TNF-*α*, IL-1*β*, and IL-6) in Patients

We examined TNF-*α*, IL-1*β*, and IL-6 concentrations in patients' serum (Figure 2). Data showed no statistical difference in pretreatment TNF-*α*, IL-1*β*, and IL-6 between groups (*P* > 0.05). Evident decreases were observed in the above three indexes in posttreatment (*P* < 0.05), and the improvement degree was more significant in OG (*P* < 0.05).

## 4. Discussion

Periarticular fractures of the shoulder are a condition including fractures of the clavicle and scapula around the shoulder joint [13]. For such fractures, conservative treatment methods, such as arm sling and spica bandages, are usually used [14]. However, the application of these traditional treatments has limitations such as poor efficacy, bone fragment movement, and nursing difficulties [15]. Therefore, it is of great practical significance to change the treatment methods to improve the curative effect and safety in view of various hindrances in the past treatment of such fractures.

BCFS is a novel type of clamp-rod internal fixation device that is commonly used for the fixation of upper and lower extremity or pelvic fractures [16]. Previous biomechanical and clinical analysis shows that BCFS is also effective in treating long bone fractures [17]. BCFS has certain advantages in treating periarticular fractures of the shoulder, as it has little contact with the bone surface and can minimize the damage of periosteal perfusion [18]. A total of 100 subjects were enrolled in this study and were assigned to two groups (CG and OG) based on the difference in treatment methods. CG was treated with plate fixation, while OG was treated with BCFS. The results showed a statistically higher ORR in OG compared with CG (96.00% vs. 80.00%), which suggested that BCFS treatment was helpful to improve the curative effect of such patients. Then, we recorded patients' clinical indices such as fracture healing time and found faster fracture healing and shorter LOS in OG, suggesting higher recovery efficiency in patients with periarticular fractures of the shoulder treated with BCFS. In the biomechanical study of BCFS, Wang et al. [19] pointed out that BCFS could more firmly fix the fracture and maintain the stability of the fracture end, with a positive effect on the fracture healing of patients. Shoulder function was also assessed in this study using the CMS, one of the most commonly used tools, which includes the measurement of patients' mobility, pain, power, and ADL [20]. The data showed significantly better shoulder joint function improvement in OG at 6 months postoperatively, which was mutually verified with the efficacy of this procedure and the results of clinical indices. In the study of Niu et al. [21] on clinical application of BCFS in mid-clavicular fractures, the postoperative CMS score is similar to that of this study.

The incidence of complications such as healing deformity, bleeding, and infection was also compared, and the results revealed a statistically lower incidence in OG as compared to CG (4.00% vs. 22.00%), which indicated that BCFS was safer than plate fixation in the treatment of periarticular fractures of the shoulder. Wang et al. [17] applied BCFS to treat femoral fractures, and no postoperative implant fracture, wound infection, or other serious complications occurred, similar to our research results. Finally, we detected three serum proinflammatory markers, namely, TNF-*α*, IL-1*β*, and IL-6; the three are highly correlated with patients' immune response, and their increased concentrations will reduce patients' immune function [22]. The results showed that postoperatively, the three indexes in OG were significantly lower than those before treatment and CG, which suggested that BCFS had an inhibitory effect on the inflammatory response of patients with periarticular fractures of the shoulder. In the study of inflammatory cytokines after fracture, Wahl et al. [23] pointed out that the proinflammatory environment brought about by inflammatory factors such as TNF-*α*, IL-1*β*, and IL-6 may be the catalyst for the development of postfracture complications; so, the inhibition of the inflammatory response of patients plays an auxiliary role in reducing complications.

Although this study confirmed that BCFS applied to patients with periarthritis of periarticular fractures of the shoulder can contribute to accelerated fracture healing, faster recovery of shoulder function, better improvement of serum inflammatory indicators, and reduction of complication rate, there are still some deficiencies. Considering the limited number of cases (*n* = 100) included, we need to expand the sample size to improve the accuracy of the research results. Second, fracture healing is a slow process, while there is no follow-up investigation in the study design. So, increasing the follow-up of 8-24 months after surgery is needed to more intuitively track patients' recovery. The above two shortcomings will be addressed in future research.

## 5. Conclusion

Conclusively, BCFS is more effective, safer, and simpler in operation than plate fixation in treating periarticular fractures of the shoulder, with good clinical application potential and value for clinical use.

## Figures and Tables

**Figure 1:** Shoulder joint function score of patients with periarticular fractures of the shoulder. Shoulder function (Constant-Murley Scale) scores of patients in both groups before and 6 months after operation. Note: ^∗∗^*P* < 0.01.

**Figure 2:** Serum inflammatory indicators (TNF-*α*, IL-1*β*, and IL-6) in patients. (a) TNF-*α* levels before and after treatment in the two groups. (b) IL-1*β* levels before and after treatment in the two groups. (c) IL-6 levels before and after treatment in the two groups. Note: ^∗∗^*P* < 0.01.

**Table 1:** Baseline data of patients with periarticular fractures of the shoulder (*n* (%), mean ± SEM).

Factor	*n*	Control group (*n* = 50)	Observation group (*n* = 50)	*χ* ^2^/*t*	*P*
Sex				0.372	0.542
Male	59	28 (56.00)	31 (62.00)		
Female	41	22 (44.00)	19 (38.00)		
Age (years old)				1.073	0.300
<35	37	21 (42.00)	16 (32.00)		
≥35	63	29 (58.00)	34 (68.00)		
Average age (years old)	100	37.06 ± 9.14	37.32 ± 8.47	0.148	0.883
Cause of injury				6.458	0.091
Car accidents	40	22 (44.00)	18 (36.00)		
Falls	27	11 (22.00)	16 (32.00)		
Crushes	17	12 (24.00)	5 (10.00)		
Others	16	5 (10.00)	11 (22.00)		
Education level				0.360	0.548
Technical secondary school or above	49	23 (46.00)	26 (52.00)		
Technical secondary school below	51	27 (54.00)	24 (48.00)		
Drinking history				1.051	0.305
No	39	22 (44.00)	17 (34.00)		
Yes	61	28 (56.00)	33 (66.00)		
Residence				0.877	0.349
Urban areas	76	40 (80.00)	36 (72.00)		
Rural areas	24	10 (20.00)	14 (28.00)		
Marital status				0.735	0.391
Single	32	14 (28.00)	18 (36.00)		
Married	68	36 (72.00)	32 (64.00)		

**Table 2:** Clinical indices of patients with periarticular fractures of the shoulder.

Groups	*n*	Fracture healing time (weeks)	Length of hospital stay (d)
Control group	50	13.00 ± 1.59	12.88 ± 1.30
Observation group	50	10.40 ± 1.29	9.50 ± 0.95
*t* value	—	8.979	14.843
*P* value	—	<0.001	<0.001

**Table 3:** Curative effect of patients with periarticular fractures of the shoulder (*n* (%)).

Groups	*n*	Marked effectiveness	Effectiveness	Ineffectiveness	Total effective rate (%)
Control group	50	22 (44.00)	18 (36.00)	10 (20.00)	40 (80.00)
Observation group	50	31 (62.00)	17 (34.00)	2 (4.00)	48 (96.00)
*χ* ^2^ value	—	—	—	—	6.061
*P* value	—	—	—	—	0.014

**Table 4:** Incidence of complications in patients with periarticular fractures of the shoulder (*n* (%)).

Categories	Control group (*n* = 50)	Observation group (*n* = 50)	*χ* ^2^ value	*P* value
Healing deformity	2 (4.00)	1 (2.00)	—	—
Blood ooze	7 (14.00)	1 (2.00)	—	—
Infection	2 (4.00)	0 (0.00)	—	—
Total incidence	11 (22.00)	2 (4.00)	7.162	0.007

## Data Availability

The labeled dataset used to support the findings of this study are available from the corresponding author upon request.
